RETRACTED

# Effects of bilateral Pecto-intercostal Fascial Block for perioperative pain management in patients undergoing open cardiac surgery: a prospective randomized study

**DOI:** 10.1186/s12871-021-01391-w

**Published:** 2021-06-22

**Authors:** Yang Zhang, Haixia Gong, Biming Zhan, Shibiao Chen

**Affiliations:** 1 Department of Anesthesiology, First Affiliated Hospital of Nanchang University, 17 Yong wai zheng Street, Nanchang, 330006 Jiangxi China; 2 Department of cardiology, The second Affiliated Hospital of Nanchang University, NO.1 minde Street, Nanchang, 330006 Jiangxi China

**Keywords:** Pecto-intercostal Fascial Block, Insulin resistance, The length of hospital stay, Sufentanil, Open cardiac surgery

## Abstract

**Background:**

Open cardiac surgical patients may experience severe acute poststernotomy pain. The ultrasound-guided Pecto-intercostal Fascial Block (PIFB) can cover anterior branches of intercostal nerves from T2 to T6. The aim of this study was to investigate the effect of bilateral PIFB in patients undergoing open cardiac surgery.

**Methods:**

A group of 108 patients were randomly allocated to either receive bilateral PIFB (PIFB group) or no nerve block (SALI group). The primary endpoint was postoperative pain. The secondary outcome measures included intraoperative and postoperative sufentanil and parecoxib consumption, time to extubation, time to first feces, length of stay in the ICU and the length of hospital stay. Insulin, glucose, insulin resistance and interleukin (IL)-6 at 1, 2, 3 days after surgery were mearsured. The homeostasis model assessment (HOMA-IR) was used to measure perioperative insulin resistance.

**Results:**

The PIFB group reported significantly less sufentanil and parecoxib consumption than the SALI group. Compared to the PIFB group, the SALI group had higher Numerical Rating Scale (NRS) pain scores at 24 h after operation both at rest and during coughing. The time to extubation, length of stay in the ICU and length of hospital stay were significantly decreased in the PIFB group compared with the SALI group. The PIFB group had a lower insulin, glucose, IL-6, HOMA-IR level than the SALI group 3 days after surgery.

**Conclusion:**

Bilateral PIFB provides effective analgesia and accelerates recovery in patients undergoing open cardiac surgery.

**Trial registration:**

This study was registered in the Chinese Clinical Trial Registry (ChiCTR 2000030609) on 08/03/2020.

## Background

There are more than 1.5 million patients worldwide undergoing open heart surgery every year [1]. Open cardiac surgical patients may experience severe acute poststernotomy pain, which is associated with persistent postsurgical pain at 1 year in 35% of patients [2]. Poststernotomy pain leads to decreased patient satisfaction, delirium, cardiovascular complications (hypertension, tachycardia, arrhythmias), hyperglycemia and respiratory complications (bronchial secretion stasis, atelectasis and pneumonia) [3]. Patient-controlled analgesia with intravenous opioids is most commonly used to alleviate pain after cardiac surgery, but opioids can cause adverse effects including delayed tracheal extubation, respiratory depression, sedation, ileus, nausea, vomiting, immunosuppression, cough suppression, drowsiness and increased risk of chronic pain [4].

RETRACTED

Epidural anesthesia (EA) and paravertebral blocks can provide effective analgesia with earlier extubation and reduced opioid use in cardiac surgical patients [5], but adverse effects related to pneumothorax, injury to the spinal cord, sympathectomy-induced hypotension, devastating epidural hematoma after full heparinization have limited the application of them in cardiac surgical patients [5]. So an ultrasound-guided peripheral nerve block technique may be advantageous in patients undergoing cardiac surgery.

The ultrasound-guided Pecto-intercostal Fascial Block (PIFB) has been advocated by some researchers for cardiac surgery [6]. Garcia et al proposed that PIFB has the advantages of avoiding pneumothorax and vascular injury compared with the transversus thoracis muscle plane (TTMP) block in cardiac surgical patients [7].

Therefore, bilateral PIFB blocks may provide effective analgesia in patients undergoing open cardiac surgery. The aim of this study was to assess whether bilateral PIFB provide effective analgesia and promote rapid recovery after open cardiac surgery.

## Methods

This study was approved by the ethics committee of First Affiliated Hospital of Nanchang University and written informed consent was obtained from all subjects participating in the trial. Then it was registered in the Chinese Clinical Trial Registry (registration number ChiCTR 2000030609). Our study adheres to CONSORT guidelines.

This double-blind, randomized, controlled study was performed on patients between the age groups of 20 and 70 years undergoing valve replacement surgery through median sternotomy with American Society of Anesthesiologists physical status III/ IV. Criteria for exclusion in our trial was as follows: emergency surgery, an allergy to local anesthetics, congestive heart failure, hepatic or renal failure, a history of drug abuse or chronic pain, psychiatric problems, secondary surgery, inability to provide informed consent. The patients enrolled in our study were randomly divided into two groups: PIFB group receiving bilateral PIFB with 0.4% ropivacaine and SALI group receiving the same block with saline.

RETRACTED

### Surgery and anesthesia

Inside the operating room, electrocardiography, invasive arterial blood pressure, oxyhemoglobin saturation, end-tidal carbon dioxide, central temperature, central venous pressure and urine output were continuously monitored in all patients in our study intraoperatively. Anesthetic induction was performed with midazolam 0.05 to 0.1 mg/kg, sufentanil 0.8 to 1 μg/kg, etomidate 0.3 mg/kg and rocuronium 0.6 mg/kg for tracheal intubation. The maintenance of anesthesia was achieved with sufentanil, propofol and rocuronium according to the clinical needs following induction in both groups, and the BIS was maintained between 45 and 55 in all patients. Intravenous sufentanil with patient-controlled analgesia was used to perform postoperative analgesia and 20 mg parecoxib was injected i.v. at 6 h intervals as a supplementary analgesic according to the demands of the patients. All surgeries were performed by the same group of surgeons in our trial. After the operation, the patients were sent to the cardiac surgery ICU as scheduled.

### Randomization and blinding

After patients entered the operating room, randomization was performed at the post anesthesia care unit to either PIFB group or SALI group using a computer- generated random number table and was kept in sealed envelopes by a biostatistician. The envelopes were opened by another researcher and he prepared the normal saline or 0.4% ropivacaine according to the group allocation. The anesthesiologist administered bilateral PIFB and he had no knowledge of whether the fluid is ropivacaine or saline after induction of anesthesia. Postoperative visitors were blinded to group allocation. This was a double-blind, randomized, controlled study.

### Ultrasound-guided PIFB

The PIFB was performed in a supine position using high-frequency linear ultrasound probe (Mindray, Shenzhen, China). The probe was placed at 2 cm lateral from sternum and parallel to the sternum, then we could find the pectoralis major muscle, the external intercostal muscle, the costal cartilage, the pleura and the lungs. Pecto-intercostal fascial plane was located between the pectoralis major muscle and the external intercostal muscle or the costal cartilage. A 20-gage, 70 mm needle (Tuoren, Henan, China) was placed under the pectoralis major and above the external intercostal muscle with in-plane approach and a test bolus of saline (2 mL) was injected to determine that the tip has been placed in the correct fascial layers. Finally, 20 ml of 0.4% ropivacaine was injected to this plane in two locations, over 2nd and 4th rib. The method on the other side of the PIFB was the same. All PIFBs were completed by the same skilled anesthesiologist within 20 min and were completed in the operating room before anesthesia induction.

RETRACTED

### Clinical and biochemical parameters

The primary outcome measures of our study were postoperative pain at 2,4,8,16,24, and 48 h after extubation at rest and exercise (defined as pain experienced during coughing) and analgesia requirements (sufentanil and parecoxib consumption). Secondary outcomes included time to drain removal, time to extubation, time to first feces, length of stay in the ICU, incidence of postoperative nausea and vomiting (PONV), the length of hospital stay, and possible complications such as ropivacaine allergy, hematomas, infections. Postoperative pain was measured using the Numerical Rating Scale (NRS) score from 0 (no pain) to 10 (worst severe pain).

Interleukin (IL) IL-6, insulin, glucose and insulin resistance were measured at before induction of anesthesia,1, 2, 3 days after surgery. Whole blood was immediately centrifuged at 1500 rpm for 20 min to separate the plasma. Then it was frozen at − 70 °C for subsequent analysis. Insulin resistance was assessed by the homoeostasis model assessment, that is, HOMA-IR = blood glucose (mmol/l) × blood insulin (munits/ml)/22.5.

### Statistical analysis

The authors calculated the patient sample size of our trial on the basis of a pilot study (*n* = 11 patients in per group), which compared the primary endpoint of the postoperative pain scores. An estimated sample size of 45 patients in each group were needed with a type I error of α = 0.05, a type II error of β = 0.1 and a power of 90%. We finally included 20% more patients for analysis to compensate for possible dropout in our trial (*n* = 54 in each group).

Statistical analysis was performed using SAS software (version 9.1.3, North Carolina, USA). The continuous data were expressed as the mean and standard deviation, whereas the qualitative data were expressed as the frequency and percentage. The Kolmogorov-Smirnov test was used to assess the normality of the continuous data. Student’s t test was used to assess the intergroup differences with normal distribution, whereas the WilcoxonMann-Whitney test was used to assess the differences in the non-normally distributed data. The Chi-square or Fisher’s exact test were used to analyze categorical data. Biochemical data were evaluated by ANOVA for repeated measurements and Scheffe method is also used for these data. A probability value of less than 5% was considered significant.

## Results

A total of 108 patients were randomized in our trial. Of the enrolled patients, 3 had redo surgery,4 refused blood collection after surgery,3 had postoperative delirium. Ultimately, date for 98 patients were finally analyzed with 49 in each group (Fig. 1). Baseline characteristics showed no statistically significant differences between PIFB group and SALI group (Table 1).

RETRACTED

**Fig. 1:** Patient flow diagram

**Table 1:** Demographic data and surgical procedures

	PIFB group (*n* = 49)	SALI group (*n* = 49)	*P*-value
Age (years)	47.5 ± 18.9	45.6 ± 19.8	0.73
Body mass index (kg/m^2^)	22.1 ± 3.5	21.3 ± 3.8	0.57
ASA classification (III/ IV)	26/23	25/24	0.59
Duration of surgery (min)	169.8 ± 39.5	175.6 ± 35.9	0.69
Size of incision (cm)	18.6 ± 3.3	17.8 ± 4.5	0.67
Cardiopulmonary bypass time (min)	76.5 ± 23.5	73.3 ± 21.5	0.57
Intraoperative bleeding volume (ml)	657.6 ± 283.9	702.8 ± 252.3	0.78
Intraoperative urine output (ml)	895.7 ± 278.4	912.5 ± 223.4	0.65
Sex (male/female)	23/26	21/28	0.67
Procedure			0.39
Mitral valve replacement	22	25	
Aortic valve replacement	27	24	

NRS pain scores were significantly lower in PIFB group compared with SALI group at 2, 4, 8 and 24 h after extubation both at rest and during coughing, and had no differences at 48 h after extubation (Figs. 2, 3). The PIFB group reported significantly decreased intraoperative and postoperative sufentanil requirement, postoperative parecoxib consumption in comparison to SALI group (Table 2). Time to extubation, length of stay in the ICU and the length of hospital stay were significantly decreased in the PIFB group (Table 2). There were no significant differences between the groups in terms of the time to first feces, incidence of PONV and the time to drain removal (Table 2). There were no complications related to PIFB in our study.

**Fig. 2:** Pain intensity at rest after extubation which was measured using the verbal numerical scale (NRS) score. * *P* < 0.05 considered statistically significant

**Fig. 3:** Pain intensity at movement after extubation which was measured using the verbal numerical scale (NRS) score. * *P* < 0.05 considered statistically significant

**Table 2:** Intra- and postoperative clinical outcomes

	PIFB group (*n* = 49)	SALI group (*n* = 49)	*P*-value
Intraoperative sufentanil consumption (μg)	118 ± 32	76 ± 10	< 0.01
Postoperative sufentanil consumption (μg)	108 ± 30	62 ± 15	< 0.01
Parecoxib consumption (mg)	60 ± 20	120 ± 40	< 0.01
Time to extubation (h)	9.7 ± 3.5	2.7 ± 1.8	< 0.01
Time to drain removal (h)	33 ± 8	30 ± 9	0.41
Length of stay in the ICU (h)	27 ± 11	17 ± 5	< 0.05
Incidence of PONV (%)	5(10.2)	7(14.3)	0.54
Time to first feces (h)	42 ± 16	39 ± 11	0.43
Length of hospital stay (h)	208 ± 23	175 ± 15	< 0.05

*P* < 0.05 considered statistically significant

There were no significant differences in the levels of insulin, glucose, IL-6, HOMA-IR between the PIFB group and the SALI group at base value. The PIFB group had a lower blood glucose level than the SALI group 3 days after operation (Table 2). Postoperatively, insulin, IL-6, HOMA-IR levels increased, and the SALI group had a higher degree than the PIFB group at 1, 2, 3 days after surgery (Table 3).

RETRACTED

**Table 3:** Measures of blood markers and insulin resistance

	Baseline	1 day after surgery	2 days after surgery	3 days after surgery
Insulin	(units/l)			
SALI group	11.56 ± 1.47	18.57 ± 4.32^*^	17.62 ± 3.21^*^	16.53 ± 1.68^*^
PIFB group	11.29 ± 1.57	13.22 ± 3.11^*^	13.13 ± 2.15^*^	12.59 ± 1.36^*^
Glucose	(mmol/l)			
SALI group	4.17 ± 2.12	6.67 ± 3.28^*^	6.37 ± 2.86^*^	6.12 ± 1.99^*^
PIFB group	4.21 ± 2.07	5.63 ± 1.65^*^	5.53 ± 1.47^*^	5.23 ± 1.37^*^
HOMA-IR				
SALI group	2.14 ± 0.57	5.50 ± 0.89^*^	4.99 ± 0.62^*^	4.49 ± 0.71^*^
PIFB group	2.11 ± 0.59	3.31 ± 0.57^*^	3.23 ± 0.56^*^	2.93 ± 0.47^*^
IL-6 (pg/ml)				
SALI group	65.15 ± 7.65	98.29 ± 9.89^*^	95.29 ± 7.87^*^	90.37 ± 6.98^*^
PIFB group	66.27 ± 6.47	83.41 ± 7.24^*^	81.62 ± 6.54^*^	78.21 ± 7.82^*^

^*^P < 0.05; *P* < 0.05 considered statistically significant

## Discussion

The present study demonstrated that the use of ultrasound-guided PIFB could reduce postoperative insulin resistance, systemic inflammation, the perioperative sufentanil consumption, dosage of postoperative parecoxib and provide effective analgesia in patients undergoing valve replacement surgery. Furthermore, these results might be the basis for reducing time to extubation, length of stay in the ICU and length of hospital stay after surgery.

The PIFB provided effective analgesia for breast surgery [8], sternal fracture pain [9], rib cage pain in ICU patients [10] and the subcutaneous-implantable cardioverter defibrillator system implantation [11].What’s more, there are some reports describing PIFB for thymectomy via median sternotomy [12, 13] and cardiac surgery [6]. To the best of our knowledge, this is the first double-blind, randomized, controlled trial to identify that bilateral PIFB provides effective perioperative pain relief in patients undergoing open cardiac surgery. Transversus thoracic muscle plane (TTMP) block was also a novel regional analgesic technique and could be used in cardiac surgery [14]. There are several reasons why PIFB could be an alternative to TTMP block [7, 15]. Firstly, transversus thoracic muscle is often very thin, difficult to visualize under ultrasound and located close to the pleura [16]. This leads to a higher risk of pneumothorax in the TTMP block. Secondly, the internal mammary artery and vein pass through the interfascial plane and the needle point is on this plane when blocking. Therefore TTMP block is at risk for vascular laceration. Thirdly, coronary artery bypass grafting could have tissue disruption in the TTMP due to artery harvest and it would affect the spread of local anesthetic [17]. In these patient, PIFB would be a better choice in open cardiac surgery.

RETRACTED

Sufentanil was most commonly used in cardiac surgery with hemodynamic stability and effective postoperative analgesia [18], but sufentanil could cause adverse effects including respiratory depression, sedation, ileus, nausea, vomiting, drowsiness, increased ICU stays [19]. In the present study, the authors revealed that the utility of bilateral PIFB decreased perioperative sufentanil dosage without adverse events because of better pain control. The mean time to extubation was significantly lower in PIFB group and the difference probably was caused by the use of a minimal amount of sufentanil. The decrease of length of stay in the ICU was associated with good analgesic effect of bilateral PIFB in open cardiac surgery, significant reduction of sufentanil dosage and early extubation after operation. Therefore, a minimal amount of sufentanil in PIFB group was an important part of the enhanced recovery of open cardiac surgery.

Patients undergoing open cardiac surgery experienced severe and prolonged postoperative pain, especially at the median sternotomy site [20]. Poorly controlled poststernotomy pain led to decreased patient satisfaction, increased rates of delirium, hemodynamic instability, pulmonary complications and increased rates of delirium [3]. Our trial demonstrated that bilateral PIFB provided effective perioperative analgesia for cardiac surgery patients both at rest and during coughing. Moreover, sufentanil and parecoxib consumption was significantly lower in the PIFB group compared to the SALI group during the 24 h after surgery. PIFB is arguably less invasive and risk than thoracic epidural, paravertebral nerve block or TTMP block with serious complications like pneumothorax, vascular laceration and epidural or spinal hemorrhage and hematoma. So ultrasound-guided PIFB was a novel, effective, promising, and safe regional analgesic technique in patients undergoing cardiac surgery and should be widely used.

Cardiopulmonary bypass and the great trauma of sawing the sternum would make cardiac patients have severe postoperative insulin resistance and systemic inflammation [21]. Postoperative insulin resistance was associated with poor outcomes in cardiac patients including increased in the frequency of infections, morbidity and mortality, delayed healing and duration of hospital stay [22, 23]. In the present study, we also found the efficiency of PIFB for the control of hyperglycemia and insulin resistance in elective open cardiac surgery. The reduction of insulin resistance is associated with a decreased inflammatory mediator release. So, the difference of postoperative insulin resistance is the main reason for the difference of IL-6 between the two groups in our study. Reduced postoperative insulin resistance and inflammatory response might be the basis for good clinical outcome in PIFB group.

RETRACTED

Finally, bilateral PIFB in patients undergoing cardiac surgery decreased perioperative sufentanil and parecoxib dosage, provided effective analgesia, reduced postoperative insulin resistance and systemic inflammation, caused earlier extubation and exit from the ICU, and these results were the basis for reducing the length of hospital stay.

This study has some limitations. The concentration and volume of the PIFB used in our trial was based on previous research. In further study, the optimum volume and concentration of the PIFB should be evaluated. Continuous PIFB may provide persistent postoperative analgesia in cardiac surgery, but our trial did not use this technique. Therefore, the utility of continuous PIFB should be further studied. Effective postoperative acute pain relief may prevent the development of chronic pain [24]. But we didn’t follow up until 1 year after the operation. In addition, our study only included patients undergoing valve replacement surgery and the impact on other patients undergoing open heart surgery needs further study.

## Conclusions

Our study found that the use of ultrasound-guided PIFB could reduce postoperative insulin resistance, systemic inflammation, the perioperative sufentanil consumption, dosage of postoperative parecoxib and provide effective analgesia in patients undergoing open cardiac surgery. Furthermore, these results might be the basis for reducing time to extubation, length of stay in the ICU and length of hospital stay after surgery.

## Data Availability

The datasets used during the current study are available from the corresponding author on reasonable request.

## Abbreviations

PIFB: Pecto-intercostal Fascial Block
EA: Epidural anesthesia
TTMP: Transversus thoracis muscle plane
PONV: Postoperative nausea and vomiting
NRS: Numerical Rating Scale
HOMA-IR: The homeostasis model assessment

## References

[1] Mozaffarian D, Benjamin EJ, Go AS, Arnett DK, Blaha MJ, Cushman M (2016). Executive summary:heart disease and stroke statistics-2016 update: a report from the American Heart Association. Circulation.

[2] van Gulik L, Janssen L, Ahlers S, Bruins P, Driessen AH, van Boven W, van Dongen E, Knibbe CA (2011). Risk factors for chronic thoracic pain after cardiac surgery via sternotomy. Eur J Cardiothorac Surg.

RETRACTED

[3] Huang AP, Sakata RK (2016). Pain after sternotomy - review. Braz J Anesthesiol.

[4] Fletcher D, Martinez V (2014). Opioid-induced hyperalgesia in patients after surgery: a systematic review and a meta-analysis. Br J Anaesth.

[5] Landoni G, Isella F, Greco M, Zangrillo A, Royse CF (2015). Benefits and risks of epidural analgesia in cardiac surgery. Br J Anaesth.

[6] Liu V, Mariano ER, Prabhakar C (2018). Pecto-intercostal fascial block for acute poststernotomy pain: a case report. A A Pract.

[7] Simón DG, Perez MF. Safer alternatives to transversus thoracis muscle plane block. Reg Anesth Pain Med. 2019. 10.1136/rapm-2019-100666.10.1136/rapm-2019-10066631300596

[8] Hong B, Yoon SH, Youn AM, Kim BJ, Song S, Yoon Y (2017). Thoracic interfascial nerve block for breast surgery in a pregnant woman: a case report. Korean J Anesthesiol.

[9] Raza I, Narayanan M, Venkataraju A, Ciocarlan A (2016). Bilateral subpectoral interfascial plane catheters for analgesia for sternal fractures: a case report. Reg Anesth Pain Med.

[10] López-Matamala B, Fajardo M, Estébanez-Montiel B, Blancas R, Alfaro P, Chana M (2014). A new thoracic interfascial plane block as anesthesia for difficult weaning due to ribcage pain in critically ill patients. Med Int.

[11] Droghetti A, Fusco P, Marini M, Harizai F, Scimia P (2019). Ultrasound-guided serratus anterior plane block and parasternal block in cooperative sedation for S-ICD implantation. Pacing Clin Electrophysiol.

[12] Song W, Wang W, Zhan L (2019). Perioperative analgesia during thymectomy via sternotomy : ultrasound-guided bilateralparasternal block. Anaesthesist..

[13] Jones J, Murin PJ (2020). Tsui JHOpioid free postoperatively using Pecto-intercostal Fascial Block (PIFB) with multimodal analgesia (MMA) in a patient with myasthenia gravis underwent thymectomy via sternotomy. J Clin Anesth.

[14] Zhang Y, Chen S, Gong H, Zhan B (2020). Efficacy of bilateral transversus thoracis muscle plane block in pediatric patients undergoing open cardiac surgery. J Cardiothorac Vasc Anesth.

[15] Fujii S. Transversus thoracis muscle plane block and alternative techniques. Reg Anesth Pain Med. 2019. 10.1136/rapm-2019-100755.10.1136/rapm-2019-10075531300594

[16] Ohgoshi Y, Ino K, Matsukawa M (2016). Ultrasound guided parasternal intercostal nerve block. J Anesth.

[17] Fujii S, Vissa D, Ganapathy S, Johnson M, Zhou J (2017). Transversus thoracic muscle plane block on a cadaver with history of coronary artery Bypass Grafting. Reg Anesth Pain Med.

[18] Kwanten LE, O'Brien B, Anwar S (2019). Opioid-based anesthesia and analgesia for adult cardiac surgery: history and narrative review of the literature. J Cardiothorac Vasc Anesth.

RETRACTED

[19] Lena P, Balarac N, Lena D, de la Chapelle A, Arnulf JJ, Mihoubi A, Tapia M, Bonnet F (2008). Fast-track anesthesia with Remifentanil and spinal analgesia for cardiac surgery: the effect on pain control and quality of recovery. J Cardiothorac Vasc Anesth.

[20] Thabane L, Ma J, Chu R, Cheng J, Ismaila A, Rios LP, Robson R, Thabane M, Giangregorio L, Goldsmith CH (2010). A tutorial on pilot studies: the what, why and how. BMC Med Res Methodol.

[21] Barth E, Albuszies G, Baumgart K (2007). Glucose metabolism and catecholamines. Crit Care Med.

[22] Floh AA, McCrindle BW, Manlhiot C (2020). Feeding may modulate the relationship between systemic inflammation, insulin resistance, and poor outcome following cardiopulmonary bypass for pediatric cardiac surgery. J Parenter Enter Nutr.

[23] Zhang Y, Min J (2020). Preoperative carbohydrate loading in gynecological patients undergoing combined spinal and epidural anesthesia. J Investig Surg.

[24] Kairaluoma PM, Bachmann MS, Rosenberg PH, Pere PJ (2006). Preincisional paravertebral block reduces the prevalence of chronic pain after breast surgery. Anesth Analg.

